# Application of Blurred Image Processing and IoT Action Recognition in Sports Dance Sports Training

**DOI:** 10.1155/2022/6189396

**Published:** 2022-10-12

**Authors:** Ligong Zhang, Chuanwei Ding, Dong Wu, Siwen Liu, Qingjian Zhao

**Affiliations:** ^1^China Wushu School, Beijing Sport University, Beijing 100084, China; ^2^School of Martial Arts and Performance, Capital University of Physical Education and Sports, Beijing 100091, China; ^3^Department of Physical Education, Beijing Institute of Technology, Beijing 100081, China

## Abstract

In order to process the blurred image, this study proposes to combine the blurred point functions in the invariant space into multiple blurred images and then restore them through the deconvolution operation. The PSF functions of the fuzzy invariant space are combined to obtain the fuzzy invariant space. Finally, a gradual restoration method is used to perform many blurred image processing steps. The experimental results prove that the method proposed in this study can avoid the noise introduced in the process of multiple deconvolutions, can reduce the calculation error, and can improve the recovery effect. Based on fuzzy image processing, this research studies the nature of human motion and the identification of actions in the Internet of Things, which provides new ideas and methods for recognition research. The Kinect somatosensory camera of the Internet of Things is used to capture deep images, and 20 three-dimensional points of the human skeleton structure are obtained through its SDK. Based on this, the motion characteristics of human joints were studied, and a motion resolution model suitable for the Internet of Things was proposed. The model has low complexity, simple calculation, and sorting characteristics. Based on this, this research study also uses software engineering ideas and general methods of system development to design and create sports dance management information systems and uses advanced methods such as computers and the Internet to maintain training management to achieve optimal sports training for sports dance mode and to provide information about the management of sports dance athletes training to improve efficiency and the management level.

## 1. Introduction

Aiming at the processing of blurred images, this study proposes a new method for estimating rotation blur parameters. This method first divides the rotated blurred image into different blocks (average and layer-by-layer block), makes each small block have an approximate angle and blur degree according to linear motion, and finally uses the least square method to estimate the rotation center and angle [1]. The experimental results show that due to the error of the actual value, the rotation center and the estimated angle are very small. At the same time, the errors obtained by incorrectly estimating the image from different block methods are also different, and it is necessary to select a suitable block method according to the actual situation [2]. Finally, this study uses two methods of displacement polar coordinates and improving diagonal load to carry out fuzzy image processing experiments and to obtain ideal recovery results. Based on this, this study designs a system for distinguishing actions of the Internet of Things [3]. The coordinate data of the secondary integration point were retrieved based on Kinect. According to the structure and distribution of the human skeleton, some joints and skeleton points are selected from the upper limbs, lower limbs, and the central connecting part to form about 22 sets of structural vectors [4]. Since the vector structure is not invariant in expansion and translation, the system further processes this basic data to obtain the characteristics of the action. Finally, 20 sets of angles and 4 sets of modulus ratio information are selected to form a 24-dimensional vector to represent the characteristics of one frame [5]. Any action composed of *n* frames is a continuous static assumption, so the system can use 24 n-dimensional vectors to design actions. In addition, the design structure of the sports dance training management information system has also been established [6].

The purpose of the system is to determine the optimal mode of sports training and complete the collection, storage, processing, and transmission of raw information of athletes in sports dance training, as well as information about coaches, training plans, influence training, and related sports dance training [7]. The system can store and retain data about the sports dance training process, can quickly and accurately perform classification and query information, can effectively obtain training information, and can search for training information according to different conditions [8]. Integrating modern information technology into the management of sports dance training can help managers and coaches. Use advanced technologies such as computers and networks to promote training management and information and automatic management of sports dance training, thereby improving efficiency and management levels [9].

## 2. Related Work

The literature introduces the overall scheme of a knowledge-based exercise-assisted training. The framework has four main modules, namely, domain knowledge, trainees, performance analysis, and management. The domain knowledge module is a digital representation of the exercise content of the sport, improvement instructions, skill indicators, and more known in the sport [10]. The literature introduces some shortcomings of common methods in image restoration algorithms. In view of the shortcomings of the traditional Wiener filtering algorithm, an improved traditional Wiener filtering algorithm was developed [11]. The data entropy function is introduced to allow secondary filtering of Wiener images, and experiments show that the algorithm can effectively restore unfocused blurred images [12]. The literature introduces the significance and importance of recognizing human actions, analyzes the ability of applying deep images to recognize actions, and provides basic research ideas for this article [13]. The literature introduces the main technology and architecture of action recognition and focuses on the methods of extracting action forms and selecting various technical details of action recognition. The literature introduces the BP neural network, which analyzes the data obtained from the neural network and uses the test data to test the BP classification algorithm. The trained network parameters are then saved and are named as VS [14]. Finally, six different operations were implemented in the VS2010 software environment for classification and identification.

## 3. Blurred Image Processing and IoT Motion Discrimination Algorithm Model

### 3.1. Blurred Image Processing Technology

Image noise may interfere with signal processing, and it is ubiquitous in the field of image acquisition and processing. Therefore, people often use probability statistics to describe it.

Noise characteristics: noise is usually a signal of image degradation (grayscale), and specific statistical characteristics (such as mean and variance) are usually used to describe noise characteristics.

Noise source: the noise source in the image is very wide. Noise will inevitably be introduced during image capture and transmission. For example, when collecting images, the amount of light and temperature in the CCD will affect the signal-to-noise ratio of the captured image. When transmitting images, factors such as the quality of the transmission equipment and atmospheric interference may also interfere with the images.

Noise is generally divided into two types, namely, the additive noise model and the multiplicative noise model.

#### 3.1.1. Additive Noise Model

(1) $$\begin{array}{c} g\left(x,y\right)=f\left(x,y\right)+n\left(x,y\right)\text{.} \end{array}$$

The output waveform of the signal affected by additive noise is the superposition state of the input signal and the noise term, and its characteristic is that the magnitude of the noise is not affected by the magnitude of the input signal.

#### 3.1.2. Multiplicative Noise Model

(2) $$\begin{array}{c} g\left(x,y\right)=f\left(x,y\right)\left[1+n\left(x,y\right)\right]=f\left(x,y\right)+f\left(x,y\right)n\left(x,y\right)\text{.} \end{array}$$

The noise multiplication will affect the output signal on both sides. The first part is the input signal of the additive noise model, and the second part is different from the additive noise model in terms of noise. It is no longer connected to the input signal, but is determined by the size of the input signal. Therefore, the multiplicative noise model has the following characteristics: as the input signal increases, the noise term also increases. This activity is difficult to calculate and analyze. In practical applications, if the input signal does not change much, then the multiplicative noise model is always evaluated as an additional processing noise model.

(3) $$\begin{array}{c} m=\underset{z_{i}\in S}{\sum }z_{i}p\left(z_{i}\right)\text{,}\\ \sigma^{2}=\underset{z_{i}\in s}{\sum }{\left(z_{i}-m\right)}^{2}p\left(z_{i}\right)\text{,} \end{array}$$

where *z*_*i*_ is the gray value of the *s* pixel and *p*(*z*_*i*_) is the value of the corresponding normalized histogram. The closest PDF can be adjusted according to the shape of the histogram of the auxiliary image *s*, and then, the mean and variance can be used to solve the necessary *a* and *b*.

In the spatial domain, the image is usually expressed as the gray value of each position in a simple and clear way. In many practical applications, after transforming complex spatial problems into a frequency domain, they will become simpler. Frequency domain processing not only helps to capture the image shape but also helps to enhance the understanding and analysis of the concept of image information, thereby helping to solve problems.

Suppose that the continuous function *f*(*x*) is sampled at *N* equidistant points to obtain the discretized function *f*(*n*) (*n* = 0,1, ..., *N* − 1), which is transformed into the discrete Fourier dimension represented as a positive transformation as

(4) $$\begin{array}{c} F\left(u\right)=\frac{1}{N}\overset{N-1}{\underset{x=0}{\sum }}f\left(x\right)e^{-j2\pi ux/N}\text{.} \end{array}$$

In the formula *x* = 0,1, ..., and *N* − 1 are the discrete time variables and *u* = 0,1, ..., and *N* − 1 are the discrete frequency variables.

The one-dimensional discrete inverse Fourier transform is

(5) $$\begin{array}{c} f\left(x\right)=\overset{N-1}{\underset{u=0}{\sum }}F\left(u\right)e^{j2\pi ux/N}\text{.} \end{array}$$

Equations (4) and (5) produce one-dimensional discrete Fourier transform pairs.

Let *f*(*x*,*y*) mark an image of the same size as *M* × *N*; then, we get

(6) $$\begin{array}{c} F\left(u,v\right)=\frac{1}{MN}\overset{M-1}{\underset{x=0}{\sum }}\overset{N-1}{\underset{y=0}{\sum }}f\left(x,y\right)e^{-j2\pi \left(\frac{ux}{M}+\frac{y}{N}\right)}\text{,}\\ f\left(x,y\right)=\overset{M-1}{\underset{u=0}{\sum }}\overset{N-1}{\underset{v=0}{\sum }}F\left(u,v\right)e^{j2\pi \left(\frac{ux}{M}+\frac{yy}{N}\right)}\text{.} \end{array}$$

In many practical applications, the image size is always a square matrix, that is, *M* = *N*. In this case, the two-dimensional discrete Fourier transform can be simplified in the following manner:

(7) $$\begin{array}{c} F\left(u,v\right)=\frac{1}{N^{2}}\overset{N-1}{\underset{x=0}{\sum }}\overset{N-1}{\underset{y=0}{\sum }}f\left(x,y\right)e^{-j2\pi \left(\frac{ux+yy}{N}\right)}\text{,}\\ f\left(x,y\right)=\overset{N-1}{\underset{u=0}{\sum }}\overset{N-1}{\underset{r=0}{\sum }}F\left(u,v\right)e^{j2\pi \left(\frac{ux+vy}{N}\right)}\text{.} \end{array}$$

It can be seen from the abovementioned formulas that the discrete two-dimensional Fourier transform is separable. In addition, the two-dimensional Fourier transform also has translation, periodicity, symmetry, rotation, and linearity, which is equal to *F*(0, 0) of MN or the average value of *f*(*x*, *y*) and other characteristics. These properties are very important in the processing and analysis of digital images.

### 3.2. Internet of Things Action Recognition Technology

The BP algorithm uses the output layer error to estimate other layer errors directly from the output layer and then uses the error to estimate the previous layer error. In this way, the error estimates for all other layers are obtained and become the final result. The displayed error will be slowly transmitted to the input end of the network, and the input direction is opposite to the input signal. Therefore, people abbreviate this algorithm as reverse reproduction algorithm or BP algorithm. It provides training for multilayer networks in a very effective way. Over the years, the algorithm has received a lot of attention, and the BP (back propagation) neural network has become one of the most commonly used neural network models. The BP network can detect many mapping relationships in the input-output model without revealing the mathematical equations that previously designed these mapping relationships. The neural network topology diagram is shown in Figure 1.

Figure 2 shows the mathematical model of the BP standard neural node. This model illustrates the three most important functions of biological neurons: weighting, summation, and transmission.

In Figure 2, *x*_1_, *x*_2_,...,*x*_*n*_ represent the inputs from neuron 1, 2, ..., *n,* respectively; *w*_*j*1_, *w*_j2_,…, *w*_*jn*_ represent neuron 1, 2, ..., *n*, neuron. The connection strength is *j*; *b*_*j*_ is the threshold; *f*(·) is the transfer function; *y*_j_ is the output of neuron *j*. The net input value *S*_*j*_ of neuron *j* is

(8) $$\begin{array}{c} S_{j}=\overset{n}{\underset{i=1}{\sum }}w_{\bar{\mu }}-b_{j}\text{.} \end{array}$$

After the net input passes through the transfer function *f* (·), the output *y*_*j*_ of neuron *j* is obtained:

(9) $$\begin{array}{c} y_{j}=f\left(S_{j}\right)=f\left(\overset{n}{\underset{i=1}{\sum }}w_{\bar{\mu }}-b_{j}\right)\text{.} \end{array}$$

The process of forming a neural network BP includes calculating (forward) data flow and propagating error signals backwards. The connection weight between the input layer and the hidden layer is *w*_*ih*_, and the connection weight between the hidden layers is layer and the output layer is *w*_ho_, hidden. The threshold of each neuron in the layer is *b*_*h*_, the standard threshold of each neuron is *b*_*o*_, the number of data samples is *k* = 1,2,3, ..., *m*, the activation function is *f*(.), and the error is calculated as

(10) $$\begin{array}{c} e=\frac{1}{2}\overset{q}{\underset{o=1}{\sum }}{\left(d_{0}\left(k\right)-yo_{o}\left(k\right)\right)}^{2}\text{.} \end{array}$$

The steps to learn the BP algorithm are as follows:

The first step is to assign a random number in the number range (−1, 1) to each connection weight from the network parameters, set the error function *e* and determine the calculated value range and the maximum number of learning *M*.

The second step is to randomly select the input sample *k* and the corresponding expected output.

(11) $$\begin{array}{c} X\left(k\right)=\left(x_{1}\left(k\right),x_{2}\left(k\right),\ldots ,x_{n}\left(k\right)\right)\text{,}\\ d_{o}\left(k\right)=\left(d_{1}\left(k\right),d_{2}\left(k\right),\ldots ,d_{q}\left(k\right)\right)\text{.} \end{array}$$

The third step is to calculate the input and output of each neuron in the hidden layer.

(12) $$\begin{array}{c} hi_{h}\left(k\right)=\overset{n}{\underset{i=1}{\sum }}w_{ih}x_{i}\left(k\right)-b_{h}h=1,2,\ldots ,p\text{,}\\ ho_{h}\left(k\right)=f\left(hi_{l}\left(k\right)\right)h=1,2,\ldots ,p\text{,}\\ yi_{o}\left(k\right)=\overset{p}{\underset{h=1}{\sum }}w_{ho}ho_{h}\left(k\right)-b_{o}o=1,2,\ldots ,q\text{,}\\ yo_{o}\left(k\right)=f\left(yi_{o}\left(k\right)\right)o=1,2,\ldots ,q\text{.} \end{array}$$

The fourth step is to calculate the partial derivative part *δ*_*b*_(*k*) of each neuron in the output layer.

(13) $$\begin{array}{c} \frac{\partial e}{\partial yi_{o}}=\frac{\partial \left(1/2\overset{q}{\underset{o=1}{\sum }}{\left(d_{o}\left(k\right)-yo_{o}\left(k\right)\right)}^{2}\right)}{\partial yi_{o}}\\ =-\left(d_{o}\left(k\right)-y_{o}\left(k\right)\right)yo_{o}^{\prime }\left(k\right)\\ =-\left(d_{o}\left(k\right)-y_{o}\left(k\right)\right)f^{\prime }\left(yi_{o}\left(k\right)\right)\\ =-\delta_{o}\left(k\right)\text{.} \end{array}$$

The fifth step is to calculate the partial derivative of the error function for each neuron in the hidden layer *δ*_*h*_(*k*).

(14) $$\begin{array}{c} \frac{\partial e}{\partial hi_{h}\left(k\right)}=\frac{\partial \left(1/2\overset{q}{\underset{o=1}{\sum }}{\left(d_{o}\left(k\right)-yo_{o}\left(k\right)\right)}^{2}\right)}{\partial ho_{h}\left(k\right)}\frac{\partial ho_{l}\left(k\right)}{\partial hi_{h}\left(k\right)}\text{,}\\ =\frac{\partial \left(1/2\overset{q}{\underset{o=1}{\sum }}{\left(d_{o}\left(k\right)-f\left(yi_{o}\left(k\right)\right)\right)}^{2}\right)}{\partial ho_{h}\left(k\right)}\frac{\partial ho_{h}\left(k\right)}{\partial hi_{h}\left(k\right)}\text{,}\\ =\frac{\partial \left(1/2\overset{q}{\underset{o=1}{\sum }}\left(d_{o}\left(k\right)-f{\left(\overset{p}{\underset{h=1}{\sum }}w_{h}ho_{h}\left(k\right)-b_{o}\right)}^{2}\right)\right)}{\partial ho_{h}\left(k\right)}\frac{\partial ho_{h}\left(k\right)}{\partial hi_{h}\left(k\right)}\text{,}\\ =-\overset{q}{\underset{o=1}{\sum }}\left(d_{o}\left(k\right)-yo_{o}\left(k\right)\right)f^{\prime }\left(yi_{o}\left(k\right)\right)w_{ho}\frac{\partial ho_{h}\left(k\right)}{\partial hi_{h}\left(k\right)}\text{,}\\ =-\left(\overset{q}{\underset{o=1}{\sum }}\delta_{o}\left(k\right)w_{ho}\right)f^{\prime }\left(hi_{l}\left(k\right)\right)\text{,}\\ =-\delta_{l}\left(k\right)\text{.} \end{array}$$

The sixth step is to change the weights *w*_*ho*_(*k*) of the hidden layer and the output layer.

(15) $$\begin{array}{c} \Delta w_{ho}\left(k\right)=-\mu \frac{\partial e}{\partial w_{ho}}=\mu \delta_{o}\left(k\right)ho_{h}\left(k\right)\text{,}\\ w_{ho}^{N+1}=w_{ho}^{N}+\eta \delta_{b}\left(k\right)ho_{h}\left(k\right)\text{.} \end{array}$$

The seventh step is to modify the connection weight *w*_*ih*_(*k*).

(16) $$\begin{array}{c} \Delta w_{ih}\left(k\right)=-\mu \frac{\partial e}{\partial w_{ih}}=-\mu \frac{\partial e}{\partial hi_{l}\left(k\right)}\frac{\partial hi_{h}\left(k\right)}{\partial w_{ih}}=\delta_{i}\left(k\right)x_{i}\left(k\right)\text{,}\\ w_{ih}^{N+1}=w_{ih}^{N}+\eta \delta_{i}\left(k\right)x_{i}\left(k\right)\text{.} \end{array}$$

The eighth step is to calculate the global error *E*.

(17) $$\begin{array}{c} E=\frac{1}{2m}\overset{m}{\underset{k=1}{\sum }}\overset{q}{\underset{o=1}{\sum }}{\left(d_{o}\left(k\right)-y_{o}\left(k\right)\right)}^{2}\text{.} \end{array}$$

The ninth step is to determine whether the network error meets the requirements. If the specified value is reached or the number of times is greater than the specified maximum number *M*, the algorithm ends. If not, return to the third step and then enter the next learning phase.

After conducting multiple experiments, by observing the experimental results, we found that if six different actions were recognized at the same time, the recognition results of three different actions were not ideal. In order to solve this problem, this study describes a hierarchical neural network BP consistent with the classification results. The “level” here is different from the input, output, and hidden layers of the BP neural network.

## 4. Practical Application of Fuzzy Image Processing in the Optimal Mode of Sports Dance Sports Training

### 4.1. Mode Structure Design

The sports dance training management system is a computer software system used for all functions of the sports dance training team, which is used to manage and supervise training activities. According to the functions of different themes, in the design of the system, these themes are divided into five categories, namely, coaches, coaches, athletes, scientific researchers, and managers, that is, five roles trained by system users.

#### 4.1.1. Head Coach

The head coach is the director of the sports dance team and manages the team's coaching staff. The head coach is the user with the highest authority among the system users. The main functions of the head coach include creating accounts for coaches, managers, and athletes; creating accounts at the same level as him; submitting annual and weekly training plans; conducting phase tests of training plans and class hours training plans; and making competition plans.

#### 4.1.2. Coach

Coach refers to the members of the sports team's coaching staff, all coaches in the athlete's training process, including sports coaches, dance coaches, and assistant coaches. Their main task in the system is to introduce the training plan, training summary, test results, and competition information at the introductory stage. The annual training plan and competition plan are mainly made by the head coach, while the weekly training plan and training plan during class are made by all coaches.

#### 4.1.3. Athletes

Athletes refer to the athletes of the sports dance team. The athlete's account is created by the head coach or team leader. After identity verification, the athlete completes the information, checks the training plan, and sends a training summary. Athletes must undergo sports training, and the coach, team leader, and scientific research team will perform activation operations. The above operations are based on the user.

#### 4.1.4. Research Group

The researchers set up a research team that collects data on athletes' physiological and biochemical indicators during training activities and introduces them into processing and statistical systems. The right to edit and view the scientific research team is restricted by the scientific research information team.

#### 4.1.5. Manager

Together with the head of the sports team, the officers, and other members of the management staff, they are responsible for the management of sports training. They can review the team's training status through the system and play a leading role in managing the training of athletes. The manager is also responsible for managing the center personnel of the project management, senior team leaders, and other personnel who have the authority to supervise and receive the training process of the sports team. Their role is as important as the manager's. The program allows viewing of training plans, training records, competition history, and athletes' technical files in this system. They can also submit game plans, determine game goals, and edit game information.

Five different users use different permissions, perform duties, collaborate with each other, and use the sports dance management information system as a means of managing sports training to achieve more accurate and effective information transmission, thereby helping users prepare for management decisions.

### 4.2. Mode Optimization Analysis

The sports dance training management information system is a complex management information system, which is oriented to multiple levels and has been studied by many users. Basic user information is necessary for the user to continue running the system. Each user who logs in to use this system must have a unique user name and password as the basis of identity verification, and each user name corresponds to the main information and written information. Basic user information should record the user's name, age, ethnicity, and other basic information, as well as historical records such as sports experience, educational experience, and teaching experience. As the main body of system management, information about athlete users should be more detailed, and the main body of athlete information is also an important main body of the main body information management organization. The user's role is the user's authority to use the system. Managers, coaches, and athletes, in the training management process, play different roles in different activities. If they use this management information system, they can also use the information they access and the modules available. In addition to the function of identifying different users, setting role authorization can also play a security role in protecting confidential information.

The design and plan of the entire training process start from basic training to reach the peak of the athletic level until interrupting participation in training activities is the overall plan for training athletes. The entire training plan can develop an overall plan for the athlete's career to improve their ability. The entire annual training plan should include a basic preparation phase, a special improvement phase, the most competitive phase, and a competitive continuation phase. Each stage has different training tasks and training loads, and different training goals must be achieved. The multiyear training plan needs to be adjusted and improved according to the actual training situation of the athletes and the needs of the competition. Therefore, the system should be able to manage annual training plans, weekly training plans, and class hours training plans and understand different training plans for different objects. For example, to prepare the same training plan for the entire team and to prepare a unique training plan for a certain athlete, the system can view and update each training plan at any time. It is also necessary to understand the control of training and exercise load and be able to accurately record training tasks and exercise load, and it can supervise the athlete's ability to exercise, so as to rationally perfect the athlete's training tasks and exercise tasks.

After exercise, one need to evaluate the effect of exercise. Whether the effect of training meets expectations is an important feedback indicator for improving the training plan. Evaluation of the impact of training should include all aspects of physical exercise, such as physical exercise, technology, psychology, and sports intelligence. Impact assessment methods can be divided into objective assessment and subjective assessment. The purpose of the evaluation is to determine the evaluation stiffness index and use clearer data or annotations to check the effectiveness of the athlete's training. For example, under the method of judging sports dance, the flexibility of sports dance quality can obtain obvious value through endurance and technical exercise level. Tests can be organized regularly to verify the training results of athletes at a specific stage and to evaluate objective indicators of training effects. Subjective evaluation includes coach review and athlete self-evaluation. Coaches can evaluate the subject and write training abstracts, including course abstracts and stage abstracts, depending on the athlete's condition during the training process, the execution of the training plan, and the time required to reach the training goal. Athletes can also write abstracts and describe the subjects' feelings, evaluate their training, and conduct more detailed self-assessments. In short, the training impact assessment module in the sports dance management information system should allow coaches and athletes to compile training abstracts, compile and review test results, and use training impact assessment methods to develop and modify exercise methods and plans.

The purpose and results of the training competition are convincing reasons. Sports training and competition are two influential and closely related relationships. Therefore, the training management information system must integrate information transmission into all aspects of sports training and regard competitive information management as an important part. Information about the athlete's game is also an important part of the athlete's file. The main point of athletes' sports competitions is to record, organize and analyze athletes' competition information, so as to summarize experience and lessons, research and improve training methods, and improve technical levels.

### 4.3. Mode Architecture Design

The objectives of the sports dance training management information system are defined as follows.

#### 4.3.1. Information Storage

In the training process, the information storage function of the system is used to complete the collection of initial information, such as athlete information, coach information, training plan, influence and training feedback, sports dance training, competition information, and other storage categories.

#### 4.3.2. Information Processing and Transmission

The functions of various system modules are used to analyze, integrate, and process raw data and provide the results to other users in the system information chain, so as to transmit information quickly and efficiently.

#### 4.3.3. Decision Support

The information processed by the system can be provided to system users as information related to decision-making to help management system users make decisions and reflect the purpose of timely implementation of decisions and the impact of implementation.

#### 4.3.4. Automatic Control of Sports Dance Training

The development of the system will promote the computerization and automation of sports dance training management and help administrators and coaches use advanced technologies such as computers and networks to promote training management and improve efficiency and management levels. By combining the needs of analysis stage ,we divided the sports dance management information system into six modules, namely, user management module, team management module, training plan management module, result management module training, information management module, and research management module. The frame diagram of the system structure is shown in Figure 3.

The sports dance training management information system is a comprehensive management system for multilevel users. There are high requirements for the relevance and real-time creation of each link. The design of the computer network system adopts the most popular centralized and distributed processing management system today, and the software in the management information system is stored on the server and the client. The client mainly has a user interface, a local database, and basic tools for data requests. The server function basically stores many data sources, manages data, and shares data. After receiving the “request,” the server will correctly process the client's request and return the result of the network processing. The basic structure of the composition is shown in Figure 4.

### 4.4. Data Acquisition

The information sources in the system are provided by different roles in the process of managing sports dance training, as well as different information related to the training management of different branches. Due to the limited research capabilities of individuals, they can only focus on the selection of key statistical training information. After consulting many documents, conducting research and practice, and discussing with sports dance experts, the data contained in the system was finally identified as basic user information, sports team building, training plans (including annual exercises, weekly plans, and hour plans), phase plan, training summary, test phase plan, test phase results, competition plan, competition results, and data in the research index. Data contained in the system are shown in Table 1.

The data logic of the system can be represented by a data flow diagram. The data flow diagram illustrates the data flow and system processing process, links the entire process together, and accurately shows the connection mechanism between different topics. According to the management process, the data flowchart of the system is divided into the following parts (each data processing node performs data storage during data processing, so the storage legend is omitted), as shown in Figure 5.

If the user is in the actual field of view of Kinect, he can actively detect and locate the positions of 20 joint points and display the position information in the form of three-dimensional coordinates (*x*, *y*, and *z*). Kinect can identify the positions of 20 joints on the human body, and their names are shown in Figure 6.

Unlike the depth of space, the unit of the bone space coordinate system is meters. Since there is a positive correlation between human movement and changes in these joints, the data obtained help us understand movement. As shown in Figure 7, the positive direction of the *Y*-axis is upward, the positive direction of the *Z*-axis corresponds to the direction of laser radiation, and the surface faces Kinect.

In the previous introduction of Kinect's bone image capture process, it was explained that skeleton positions are a sequence of 20 vector and 4 slots, and we only need to add them. At the same time, the specified file transfer data are operated through the file stream to obtain the three-dimensional space coordinates of the aggregation point, and 20 vectors are stored in sequence. The corresponding relationship is shown in Table 2. We can use these numbers as a matrix to access the corresponding data of the common point.

The process of constructing the human body structure vector based on the extracted common point coordinates and combining the characteristics of the human body structure is called the human body vector structure, and 22 structure vectors are defined according to the system requirements. These structure vectors are divided into upper limb structure vector (4), lower limb structure vector (4), trunk structure vector (7), and connection structure vector (7). According to the rules of defining mathematical vectors, the structure of the human body is named according to the principle that the starting point is at the front end and the endpoint is at the back end. The structure of the human body vector is marked with the right elbow⟶right hand in Chinese to facilitate intuitive understanding, where “⟶” indicates the direction of the vector. There are 4 sets of vectors in the upper limbs, composed of the arms of two people.  Table 3 shows the composition and name of the vector structure at the top.

The four groups of structural vectors of the lower limbs are composed of the joint points of the human legs and the skeleton. The composition and naming of these structural vectors are shown in Table 4.

As shown in Table 5, the body vectors of these groups are used to reflect the changes in the body during the functional process. For example, upright and sitting actions must use these vectors to distinguish them from other actions.

The vector structure of the connection part also has 7 groups. The composition and name of the merge point are shown in Table 6. This part of the structure vector mainly reflects the changes in the upper torso and head and plays an important role in the definition and solution of the modulus ratio.

## 5. Conclusion

Image restoration is widely used in research fields such as remote sensing, military, and medicine. In the process of image receiving and sending, due to various factors (for example, the relative movement of the scene and the camera and the focal length of the lens), the image quality may be degraded. However, in many practical applications, there is a high demand for clear images, which requires the use of image restoration techniques to obtain images that best meet the requirements of practical applications.

Based on the analysis of fuzzy image reproduction theory, related technologies such as linear fusion, focus fusion, uniform rotation motion fusion, and multi-image fusion were discussed, and in-depth research and discussion were carried out. Based on this model, this article uses software engineering ideas and general system methods to design and develop an information system for managing sports dance training. The system can effectively store and retrieve data in the process of sports dance training, can quickly and accurately perform classification and query information, and can effectively input training information and retrieve information. Modern information technology has also been fully integrated into the management of sports dance training, which can help managers, coaches, and other personnel use advanced technologies such as computers and networks to promote training management, information, and automated management of sports dance training, thereby improving efficiency and management level.

## Figures and Tables

**Figure 1:** BP neural network topology structure diagram.

**Figure 2:** BP neuron mathematical model.

**Figure 3:** Framework diagram of the management information system for sports dance training.

**Figure 4:** C/S platform diagram.

**Figure 5:** System data flowchart.

**Figure 6:** Node location and name.

**Figure 7:** Kinect skeleton space coordinate system.

**Table 1:** Data contained in the system.

	User basic information	Sports team establishment	Training plan	Training summary	Phase test plan	Stage test results	Game plan	Competition results	Scientific research index data
Head coach	O	√ O	√ O	√ O	√ O	√ O	√ O	√ O	O
Coach	√ O	O	√ O	√ O	O	√ O	O	√ O	O
Athlete	√ O	C	O	√ O	O		O	O	
Research group	√ O	O	O	O	O	O	O	O	√ O
Manager	O	O	O	O	O	O	√ O	√ O	O

**Table 2:** Storage order of key nodes.

English name of gateway	Chinese name of the key node	Corresponding number
HIP_CENTER	Middle of hip	0
SPINE	Spine	1
SHOULDER_CENTER	Middle of the shoulder	2
HEAD	Head	3
SHOULDER_LEFT	Left shoulder	4
ELBOW_LEFT	Left elbow	5
WRIST_LEFT	Left wrist	6
HAND_LEFT	Left hand	7
SHOULDER_RIGHT	Right shoulder	8
ELBOW_RIGHT	Right elbow	9
WRIST_RIGHT	Right wrist	10
HAND_RIGHT	Right hand	11
HIP_LEFT	Left hip	12
KNEE_LEFT	Left knee	13
ANKLE_LEFT	Left ankle	14
FOOT_LEFT	Left foot	15
HIP_RIGHT	Right hip	16
KNEE_RIGHT	Right knee	17
ANKLE_RIGHT	Right ankle	18
FOOT_RIGHT	Right foot	19

**Table 3:** Upper limb structure vector.

Body parts	Structure vector English name	Structure vector corresponding to Chinese representation
Upper limbs	RightShoulder_To_RightElbow	Right shoulder ⟶ right elbow
	RightElbow_To_RightWrist	Right elbow ⟶ right wrist
	LeftShoulder_To_LeftElbow	Left shoulder ⟶ left elbow
	LeftElbow_To_LeftWrist	Left elbow ⟶ left wrist

**Table 4:** Structure vector of the lower extremity.

Body parts	Structure vector English name	Structure vector corresponding to Chinese representation
Lower limbs	RightHip_To_RightKnee	Right hip ⟶ right knee
	RightKnee_To_RightAnkle	Right knee ⟶ right heel
	LeftHip_To_LeftKnee	Left hip ⟶ left knee
	LeftKnee_To_LeftAnkle	Left knee ⟶ left ankle

**Table 5:** Torso structure vector.

Body parts	Structure vector English name	Structure vector corresponding to Chinese representation
Trunk part	ShoulderCenter_To_RightShoulder	Middle of the shoulder⟶right shoulder
	ShoulderCenter_To_LeftShoulder	Middle of the shoulder⟶left shoulder
	Spine_To_ShoulderCenter	Spine ⟶ middle of the shoulder
	Spine_To_RightShoulder	Spine ⟶ right shoulder
	Spine_To_LeftShoulder	Column ⟶ left shoulder
	Spine_To_RightHip	Spine ⟶ right hip
	Spine_To_LeftHip	Spine ⟶ left hip

**Table 6:** Connected part structure vector.

Body parts	Structure vector English name	Structure vector corresponding to Chinese representation
Connection part	Head_To_RightWrist	Head ⟶ right wrist
	Head_To_LeftWrist	Head⟶left wrist
	Spine_To_Head	Spine⟶head
	Spine_To_RightElbow	Spine ⟶ right elbow
	Spine_To_RightWrist	Spine ⟶ right wrist
	Spine_To_LeftElbow	Spine ⟶ left elbow
	Spine_To_LeftWrist	Spine ⟶ left wrist

## Data Availability

The data used to support the findings of this study are available from the corresponding author upon request.
